# Analysis on Medication Rules of Chinese Medicinal Herb Formulae in Uterine Subinvolution Treatment Based on Data Mining

**DOI:** 10.1155/2022/1752352

**Published:** 2022-03-31

**Authors:** Jianghe Luo, Ming Yang, Yuling Liu, Xinrui Han, Wei Yue

**Affiliations:** ^1^Department of Gynecology and Obstetrics, Guangzhou Women and Children's Medical Center, Guangzhou 510623, China; ^2^School of Nursing, Guangzhou University of Chinese Medicine, Guangzhou 510006, China; ^3^Department of Obstetrics, The First Affiliated Hospital, Guangzhou University of Chinese Medicine, Guangzhou 510006, China

## Abstract

**Introduction:**

Uterine subinvolution, especially the subinvolution of the placental site, can be a life-threatening disease that induces secondary postpartum hemorrhage (PPH). Chinese Herbal Medicine has been widely used to improve postpartum recovery and treat uterine subinvolution for thousands of years. Yet, there are many potential laws hidden that are worth exploring.

**Methods:**

Prescriptions treating uterine subinvolution were searched and collected to form datasets. Data mining methods including frequency analysis, cluster analysis, and association rule learning were performed to uncover the potent prescription laws of uterine subinvolution treatment.

**Results:**

A total of 803 formulae involving 249 herbs were obtained. The top 6 most frequently used herbs were *Angelicae Sinensis Radix* (Danggui), *Chuanxiong Rhizoma* (Chuanxiong), *Leonuri Herba* (Yimucao), *Persicae Semen* (Taoren), *Zingiberis Rhizoma Preparatum* (Paojiang), and *Radix Glycyrrhizae Preparata* (Zhigancao). Most of the 249 herbs were being warm in properties, sweet in tastes, and mainly distributed to liver and spleen meridian tropisms. Deficiency-tonifying herbs accounted for the most proportion and heat-clearing herbs ranked the second, followed by blood-activating and stasis-eliminating herbs. 6 clusters were generated by hierarchical clustering, and 5 of them were of clinical significance. 78 rules with support values over 0.25, confidence values over 0.8, and lift values greater than 1 were generated by association rule learning.

**Conclusion:**

The basic principles for uterine subinvolution treatment were deficiency-tonifying, heat-clearing, blood-activating, and stasis-eliminating. Herbs with warm properties, sweet tastes, and liver and spleen meridian tropisms are generally suitable. In addition, Sheng-Hua-Tang was the most frequently used formula for the treatment of uterine subinvolution, yet the dialectical prescriptions were diversified with different patterns/symptoms.

## 1. Introduction

During the postpartum period, the enlarged uterus undergoes a physiological involution of about 6 weeks to its nonpregnant condition which is called uterine involution [1]. The involution process includes the degradation and resorption of collagen [2] which represent sequential vaginal discharge (lochia) that occurs during the first week after delivery [3], the contraction of uterine smooth muscles that manifests as the gradual decrease of symphysis pubis-uterine fundus distance [4], and the repair of endometrium and blood vessels [5]. Any failure in the process of degeneration or regeneration leads to subinvolution of the uterus [6]. The causes of uterine subinvolution include uterine atony, multiparity, retention of portions of the placenta or membranes, and infections [6]. The manifestations of uterine subinvolution contain excessive or prolonged lochia, uterine tenderness, abdominal pain, abnormal uterine volume, and diameter by ultrasonographic examination [7]. Poor uterine involution, especially subinvolution of the placental site, is closely associated with secondary postpartum hemorrhage (PPH), which is the major cause of morbidity and mortality [8–11], being a life-threatening disease to women. The treatment for uterine subinvolution consists in the removal or prevention of several causes that lead to it. Basically, emptying the uterine cavity by surgery is the main treatment for the retention of the placenta or membranes. For uterine atony, uterotonic agents are the primary drugs for treatment, and the most prescribed one is oxytocin, a nonapeptide synthesized in the hypothalamus that is effective in reducing blood loss by enhancing the contraction of uterine musculature [12, 13]. Besides, methylergonovine, carboprost, and misoprostol are also functional medications for uterine contraction and are candidate drugs for the treatment of uterine subinvolution [14, 15].

In China, uterine subinvolution is also called “lochiorrhea” (Elubujue in Chinese) that was defined as vaginal blood loss lasting over 3 weeks after child-birth and postpartum abdominal pain according to The National Administration of Traditional Chinese Medicine (TCM) [16] and was firstly recorded in Jin-Gui-Yao-Lue written by Zhongjing Zhang, a famous doctor of east Han dynasty [17]. A huge number of efficient prescriptions treating uterine subinvolution were recorded and hundreds of herbs were involved in Chinese literature [18]. There might be many prescription rules hidden in that would be valuable for clinical practice. However, few such researches have been published.

Data mining, as a widely used data information processing technology through algorithms, enables researchers to deeply discover the potential laws from multidimensional data sets [19, 20]. Hence, the objective of this study was to explore the prescription regularity of Chinese herbal medicines treating uterine subinvolution and to discover new prescription rules by integrated data mining methods. First, descriptive analysis was used to study the frequency, property, taste, and meridian tropism of all herbs. Then, cluster analysis and association rule learning were employed to analyze the prescription rules. We expect that the results of this research could provide valuable guidance for clinical practitioners on the treatment of uterine subinvolution and the improvement of puerperium involution.

## 2. Materials and Methods

### 2.1. Data Source and Processing

All related articles in this study were collected from the China database of Traditional Chinese Medicine (http://cintmed.cintcm.com/cintmed/), China National Knowledge Infrastructure (CNKI) database, Chinese BioMedical Literature Database (CBM), VIP Database of Chinese Technical Periodicals (VIP), and WanFang Data (WanFang). The subdatabases in China database of Traditional Chinese Medicine include Chinese Prescription database, Database of Chinese Pharmacopeia (2005 edition), Chinese Medicine Recipe Database, Chinese Pharmacopeia clinical medication instructions, and Database of Modern application of prescriptions. All studies published before January 30, 2021, were searched. We used two heading terms to search the studies: (a) “lochiorrhea” and “subinvolution of uterus”; (b) “pharmacotherapy,” “herbal therapy,” and “integrated Chinese and Western medicine therapy.” The representing search strategy in Chinese for CBM is (“Chanhoufutong” [unweighted: extended] OR “Zigong fujiubuliang” [unweighted: extended] OR “Elubujue” [unweighted: extended] OR “Elubuzhi” [unweighted: extended]) AND (“herbal therapy”[unweighted: extended] OR “integrated Chinese and Western medicine medicine”[unweighted: extended] OR “chemotherapy”[unweighted: extended] OR “pharmacotherapy” [unweighted: extended] OR “dietary therapy” [unweighted: extended]). Including criteria are as follows: (1) literature of Chinese Medicine treatment for uterine subinvolution. Excluding criteria are as follows: (1) literature with no-listed or not indicated complete herb components, (2) review literature, (3) case reports, and (4) animal trials. The screening process of all literature was carried out by two researchers independently first and then synthesized by a third researcher. The herb names were standardized and the information of action category, properties, tastes, and meridian tropisms was complemented according to Chinese pharmacopeia (2020 edition) [21] and Chinese Materia Medica [22]. The detailed workflow diagram is displayed in Figure 1.

### 2.2. Descriptive Analysis

Descriptive analysis is a method for statistically describing the characteristics of various variables in datasets, mainly including frequency analysis, centralized trend analysis, and dispersion degree analysis. Frequency analysis for herbal medicines has been widely used to seek prescription rules and to provide the basis for clinical forecasting and decision-making [23]. It is beneficial to better understand the nature of diseases and the typical methods of prevention or treatment. To analyze the characteristics of uterine subinvolution and to explore the preference of its herbal treatment, frequency analysis was applied to study the frequency of occurrence, action category, properties, tastes, and meridian tropisms of all herbs involved. All descriptive statistics were performed in Microsoft Excel 2016.

### 2.3. Cluster Analysis

As a powerful statistical method in classifying relatively similar data, cluster analysis is frequently used for data analysis. When applied to the study of medication rules, cluster analysis can classify the seeming scattered herbs into regular groups (clusters) and reveal the potential combination regularities for prescription [24]. To discover and summarize the rational herb combinations treating uterine subinvolution, cluster analysis of the top 40 herbs was carried out by utilizing IBM SPSS Statistics 26.0. Average linkage was used as the hierarchical agglomerative clustering method, and squared Euclidean distance was chosen as the measurement method to obtain clusters [25]; the calculated values were standardized by *Z* scores and rescaled from 0 to 1 for comparison.

### 2.4. Association Rule Learning

Association rule learning is a data mining method that was created for market basket analysis to identify how discrete values cooccur within datasets [26]. To explore the combination rules for the treatment of uterine subinvolution, association rule learning of all herbs was carried out using R studio 1.4.1103 in this study. The specific use of herbs in each prescription was converted into binary variables (e.g., herbs used = 1, herbs not used = 0). The apriori algorithm was chosen to generate candidate item sets [27]. Three measurements, support, confidence, and lift were employed to select important rules. Support refers to the probability of an item set appearing in all item sets. If the support of an item set and the number of all item combinations in the data set are recorded as Support(*X*) and |*D*|, the support calculation equation of an item set is

(1) $$\begin{array}{c} \text{Support}\left(X\right)=\frac{\text{Count}\left(X\right)}{\left|D\right|}\times 100\%. \end{array}$$

The support of an association rule refers to the cooccurrence frequency of the antecedent and the consequent which represents the support of item set *X* ∪ *Y* and can be recorded as Support(*X*⟶*Y*). So, the equation is

(2) $$\begin{array}{c} \text{Support}\left(X⟶Y\right)=\frac{\text{Count}\left(X\cup Y\right)}{D}\times 100\%. \end{array}$$

Confidence is the ratio of the frequency that the antecedent and consequent items cooccur to the frequency that the antecedent item occurs individually, indicating how accurate the rule is [28]. The calculate equation is

(3) $$\begin{array}{c} \text{Confidence}\left(X⟶Y\right)=\frac{\text{Support}\left(X⟶Y\right)}{\text{Support}\left(X\right)}\times 100\%. \end{array}$$

The lift which represents the effects of the occurrence of an antecedent on the occurrence rate of the consequent is used to determine whether the rule has actual meaning. The rule has an actual effect when the lift value is greater than 1 and has no effect when the lift value is less than 1 [29]. The equation is

(4) $$\begin{array}{c} \text{Lift}\left(X⟶Y\right)=\frac{\text{Confidence}\left(X⟶Y\right)}{\text{Support}\left(Y\right)}=\frac{P\left(X\cup Y\right)}{P\left(X\right)P\left(Y\right)}. \end{array}$$

To avoid obtaining a large number of rules, the minimum threshold of support was set to 0.25, the minimum value of confidence was set to 0.8, and the minimum threshold of the lift was set to 1, respectively. Besides, to limit the number of herbs forming an association rule to 2–6, the minimum length (min len) of a rule is set to 2, and the maximum length (max len) is set to 6.

## 3. Results

### 3.1. Descriptive Analysis

#### 3.1.1. Herb Frequency

After data collection and processing, a total of 803 formulae and 249 herbs were obtained. The 249 herbs were used 7799 times in all and 40 of them were used over 48 times each.  Table 1 presents the top 40 most used herbs treating uterine subinvolution with an accumulative rate of 81.47%. According to Table 1, *Angelicae Sinensis Radix* (Danggui) was used 679 times and the rate equals 8.71%, ranking the most used herb in the treatment of uterine subinvolution. The second commonly used herb is *Chuanxiong Rhizoma* (Chuanxiong) which appeared 586 times and accounted for 7.51%. Besides, *Leonuri Herba* (Yimucao, appeared 554 times and accounted for 7.10%) were *Persicae Semen* (Taoren, appeared 509 times and accounted for 6.53%) were also high frequently used herbs, indicating the important roles of those herbs in uterine subinvolution treatment.

To more intuitively disclose the trends in the frequency of herbal usage and its inherent meaning, Figure 2 was drawn for analysis. After comparison and analysis, the frequencies of the top five most used herbs were found to be much higher than that of the rest, revealing the key role of these herbs in uterine subinvolution treatment. What's more, the frequencies of *Astragali Radix* (Huangqi), *Zingiberis Rhizoma Preparatum* (Paojiang), *Pollen Typhae* (Puhuang), and *Codonopsis Radix* (Dangshen) are similar and significantly higher than that of the posterior herbs, which reflects the high rate of use in subtraction or addition of prescriptions treating uterine subinvolution.

#### 3.1.2. Properties, Tastes, and Meridian Tropisms of Herbs

The properties, tastes, and meridian tropisms refer to the capability of herbs and are high-level summaries of the basic properties and characteristics of herbal efficacy. In the theories of TCM, diseases are all basically caused by the body's imbalance of Yin and Yang being prosperous or declining and could be classified into cold or heat syndromes. The properties of herbs are described as Four Qi, including cold, hot, warm, and cool, reflecting the tendency to affect the rise and fall of Yin and Yang and the change of cold and heat in the human body. Four Qi is one of the important concepts that explain the action properties of herbs. However, some herbs are not obvious in cold or hot tendency, which could be classified as mild in the property. Therefore, five properties were chosen for analysis in this study according to TCM theories. Tastes are the characteristics of herbs reflecting the roles in tonifying, purging, dispersing, astringing, etc. The basic tastes of herbs include pungent, sour, sweet, bitter, salty, weak, and astringent. The meridian tropisms of herbs refer to the attributes acting on different parts of the human body and could indirectly reflect the special organs or tissues related to diseases and their treatment. There were 12 different meridian tropisms selected for analysis in this study. All properties, tastes, and meridian tropisms of the 249 herbs are summarized in Figure 3. As Figure 3(a) shows, the main properties are warm (3420 times), mild (2311 times), and cold (1865 times). As shown in Figure 3(b), the main taste is sweet (4468 times), followed by bitter (3912 times) and pungent (3097 times). As shown in Figure 3(c), most of the 249 herbs are attributed to liver, spleen, and heart meridian tropisms.

#### 3.1.3. Action Category of Herbs

Chinese herbal medicines can be classified into different categories according to their special effects. Based on Chinese Materia Medica, there are 21 kinds of categories treating different TCM patterns/syndromes.  Table 2 shows the classification and proportion of all 249 herbs used in all prescriptions. As shown in Table 2, all herbs involved in this study could be divided into 19 categories, and deficiency-tonifying herbs accounted for the largest proportion (34.43%) with a frequency of 2685. Besides, blood-activating and stasis-eliminating herbs took the second place of proportion (29.98%) with a frequency of 2338. In addition, hemostatic herbs ranked third with a proportion of 12.85% and heat-clearing herbs accounted for the fourth with a proportion of 9.26%.

The percentages of the number of herbs in each category to the total (249) are shown in Figure 4. According to Figure 4, there are 41 deficiency-tonifying herbs, accounting for the largest percentage (16.5%). Besides, 38 of the 249 herbs (15.3%) belong to heat-clearing herbs and 29 (11.6%) belong to blood-activating and stasis-eliminating herbs.

### 3.2. Cluster Analysis

The dendrogram of 40 core herbs was generated by cluster analysis as shown in Figure 5. The herbs could be divided into 6 different clusters at a distance of 23. All clusters were composed of multiherbs, and 5 of them are meaningful in clinical prescription.

### 3.3. Association Rule Learning

A total of 78 rules were obtained with support values over 0.25, confidence values over 0.8, and lift values greater than 1 by association rule learning. The whole detailed rules are exhibited in Table 3. The pictorial overview of the 78 association rules is shown in Figure 6. As shown in Table 3, {*Chuanxiong Rhizoma* (Chuanxiong)} ≥ {*Angelicae Sinensis Radix* (Danggui)} and {*Angelicae Sinensis Radix* (Danggui)} ≥ {*Chuanxiong Rhizoma* (Chuanxiong)} have the highest support level of 0.72. {*Angelicae Sinensis Radix* (Danggui), *Chuanxiong Rhizoma* (Chuanxiong), *Leonuri Herba* (Yimucao), *Zingiberis Rhizoma Preparatum* (Paojiang)} ≥ {*Persicae Semen* (Taoren)} has the highest lift level with 1.52. There are eight association rules (rule 55, 72, 66, 27, 63, 51, 46, 75) consisting of *Chuanxiong Rhizoma* (Chuanxiong), *Leonuri Herba* (Yimucao), *Persicae Semen* (Taoren), *Zingiberis Rhizoma Preparatum* (Paojiang), *Angelicae Sinensis Radix* (Danggui), *Astragali Radix* (Huangqi), and *Radix Glycyrrhizae Preparata* (Zhigancao) with the highest confidence level of 1, revealing the strong correlations between those herbs and their compatible use in prescriptions treating postpartum uterine subinvolution. It could be seen from Figure 6 that herbs *Chuanxiong Rhizoma* (Chuanxiong), *Leonuri Herba* (Yimucao), *Persicae Semen* (Taoren), *Zingiberis Rhizoma Preparatum* (Paojiang), *Angelicae Sinensis Radix* (Danggui), and *Radix Glycyrrhizae Preparata* (Zhigancao) were at the center of the network graph, indicating they are the core herbs for prescriptions.

## 4. Discussion

### 4.1. The Main Characteristics for Uterine Subinvolution Treatment

This study determined functional herbal formulae for uterine subinvolution treatment by integrated methods based on frequency analysis, cluster analysis, and association rule learning. We summarized herb frequency, properties, action categories and assessed the potential prescribing rules between herbs. Our results showed that the most frequently used herbs were *Angelicae Sinensis Radix* (Danggui), followed by *Chuanxiong Rhizoma* (Chuanxiong), *Leonuri Herba* (Yimucao), *Persicae Semen* (Taoren), *Zingiberis Rhizoma Preparatum* (Paojiang), and *Radix Glycyrrhizae Preparata* (Zhigancao). The properties of these herbs were mainly being warm, mild, and cold. The tastes of these herbs were predominantly sweet and bitter. Most of these herbs were distributed to liver and spleen meridian tropisms and generally being deficiency-tonifying, heat-clearing, blood-activating, and stasis-eliminating. 5 meaningful clusters were obtained by cluster analysis. Cluster 1 was mainly prescribed for nourishing liver-spleen, cluster 2 was effective for clearing heat and regulating Qi, cluster 3 was functional at blood-activating and stasis-eliminating, cluster 4 was mainly used for hemostasis and blood replenishment, and cluster 6 was prescribed for tonifying Yang and clearing heat. 78 rules were extracted by association rule learning, and herbs *Chuanxiong Rhizoma* (Chuanxiong), *Persicae Semen* (Taoren), *Angelicae Sinensis Radix* (Danggui), *Zingiberis Rhizoma Preparatum* (Paojiang), *Leonuri Herba* (Yimucao), and *Radix Glycyrrhizae Preparata* (Zhigancao) were found to be strongly correlated, indicating that they were the basic herbs in the treatment of uterine subinvolution for clinical addition and subtraction. To better understand the results of data mining from TCM theories, the action categories of the top 40 herbs were listed in Table 4.

The basic pathogenesis of uterine subinvolution can be ascribed to blood deficiency, blood heat, and blood stasis, which usually exist simultaneously [30]. According to TCM theories, the relationship between Qi and blood can be summarized as “Qi is the general of blood and blood is the mother of Qi (气为血之帅,血为气之母)” and is mainly reflected in four aspects. (1) Blood has a nourishing effect on Qi. When blood is sufficient, Qi will flourish, and when blood is deficient, Qi will be deficient easily. (2) Qi exists in and is attached to blood, so blood deficiency will lead to Qi deficiency diseases. (3) Qi participates in and promotes the generation of blood and so Qi deficiency is easy to lead to blood deficiency diseases. (4) Qi can promote and regulate the steady movement of blood in the veins. When Qi is sufficient, blood flow is smooth. Conversely, if Qi is deficient, it cannot promote blood flow, resulting in blood stasis. From Table 2, Figure 4, and Table 4, deficiency-tonifying herbs accounted for the largest proportion and heat-clearing herbs ranked the second followed by blood-activating and stasis-eliminating herbs, indicating the principle of uterine subinvolution treatment: tonic is the main method and supplemented by heat-clearing, blood-activating, and stasis-eliminating. Tonifying herbs such as *Angelicae Sinensis Radix* (Danggui) and *Radix Glycyrrhizae Preparata* (Zhigancao) mainly targeted the liver and spleen to exert their functions. The liver storing blood and the spleen governing transportation and transformation could help to absorb, transform, and store the essence of food for body needs, which is vital for the generation of blood and Qi. Most of the frequently used herbs were being warm in properties which are effective in dispelling internal cold, enhancing and activating the vital Qi to defend the six exogenous evils. Sweet was the main taste of the 249 involved herbs and was considered owing the effects of nourishing, neutralizing, reconciling herbs, and relieving acute pain. These characteristics mentioned above indicated that herbs with warm properties, sweet tastes, and liver and spleen meridian tropisms are generally suitable for the treatment of postpartum uterine subinvolution to replenish blood-Qi, activate blood flow, and eliminate stasis.

### 4.2. The Prescription Rules for Uterine Subinvolution Treatment

Descriptive analysis showed the predominant principles for uterine subinvolution treatment and the main characteristics of herbs prescribed while cluster analysis and association rule learning further explored the specific medication rules. As Figure 5 shows, cluster 1 contained 9 herbs which are relatively frequently used in all prescriptions. Cluster 1 was the most commonly used prescription in clinical practice and had the balanced function of Qi-blood replenishing, blood-activating, and stasis-eliminating. *Herba Taraxaci* (Pugongying), *Herba Patriniae* (Baijiangcao), and *Portulaca Herba* (Machixian) in cluster 2 are all heat-clearing herbs. *Aurantii Fructus* (Zhike) has the function of Qi-regulating/activating and *Crataegi Fructus* (Shanzha) is effective in stasis-eliminating. Those two herbs together are of significant effectiveness for uterine subinvolution with abdominal pain induced by the impede of stasis and herbs in cluster 2 can be prescribed when the blood heat patterns are obvious complicated with blood stasis symptoms. Cluster 3 was comprised of 7 herbs and 5 of them are blood-activating and stasis-eliminating herbs, making it the best choice of clinical prescription when blood stasis pattern is predominant. Cluster 4 was composed of 3 Qi tonic herbs, 3 hemostatic herbs, and 1 superficies-relieving herb, which can be used in combination in uterine subinvolution patients with much lochia. Cluster 6 was composed of 9 herbs. Among them, *Dipsaci Radix* (Xuduan), *Eucommiae Cortex* (Duzhong), *Paeoniae Radix Alba* (Baishao), *Rehmanniae Radix Praeparata* (Shudihuang), and *Rhizoma Dioscoreae* (Shanyao) are all deficiency-tonifying herbs. *Rehmanniae Radix* (Dihuang), *Moutan Cortex* (Mudanpi), and *Radix Sanguisorbae* (Diyu) are all heat-clearing herbs. The compatibility of herbs in cluster 6 focuses on replenishing Yang, which is suitable for severe deficiency patterns of uterine subinvolution. In summary, Figure 7 is drawn to better elucidate the prescription regularities.

As shown in Figure 6(c), 9 herbs were involved in the 78 rules and *Chuanxiong Rhizoma* (Chuanxiong), *Persicae Semen* (Taoren), *Angelicae Sinensis Radix* (Danggui), *Zingiberis Rhizoma Preparatum* (Paojiang), *Leonuri Herba* (Yimucao), and *Radix Glycyrrhizae Preparata* (Zhigancao) were at the center which strongly correlated with each other. Those herbs were consistent with the components of cluster 1, revealing that they formed the core prescription in uterine subinvolution treatment which is similar to the famous formula Sheng-Hua-Tang (composed of *Angelicae Sinensis Radix* (Danggui), *Chuanxiong Rhizoma* (Chuanxiong), *Persicae Semen* (Taoren), *Zingiberis Rhizoma Preparatum* (Paojiang), and *Glycyrrhizae Radix Et Rhizoma* (Gancao)). In Chung et al.'s research, Sheng-Hua-Tang was used by 86.2% of postpartum women in Taiwan, being the most prescribed herbs in the puerperium period [31]. Sheng-Hua-Tang was firstly recorded in *Bamboo Grove Temple Gynecology*, the secret recipe of medical monks in Bamboo grove Temple [32]. According to TCM theories, *Angelicae Sinensis Radix* (Danggui) is the monarch herb in Sheng-Hua-Tang with blood tonifying-activating and stasis-eliminating effects. *Chuanxiong Rhizoma* (Chuanxiong) is the minister herb that is good at Qi-blood-activating and stasis-eliminating. *Persicae Semen* (Taoren) and *Zingiberis Rhizoma Preparatum* (Paojiang) are the assistant herbs that are efficient in blood-activating, stasis-eliminating, cold-dispersing, and pain-relieving. *Glycyrrhizae Radix Et Rhizoma* (Gancao) is the guide herb that acts as a harmonizing role. With the synthetic effects, Sheng-Hua-Tang is efficient in blood-activating and stasis-removing and functional at the discharge of lochia and involution of the uterus. Besides, Sheng-Hua-Tang was shown to participate in the returning of the uterus to its anteverted position [33] and to increase the contractile activity of the myometrium [34]. Modern pharmacological studies have indicated that Sheng-Hua-Tang could also reduce drug-induced uterine bleeding in medical abortion through regulating estradiol, estrogen receptor, progesterone receptor, fibronectin, laminin [35], and Th1/Th2/Th17/Treg paradigm [36].

### 4.3. Limitations

There are some limitations to our study. First, only five databases of Chinese Medicine were searched and articles published in English were not found, which may limit the applicability of our findings to some extent. Second, the dosage of herbs prescribed was deleted during data processing for the difficulties in standardizing different units. So, the clinical dosage and ratio of each herb in prescription were unclear, and future studies including the dose-effect relationship of herb combinations are still warranted. Third, although some of the articles included in this study were performed for the specific patterns of uterine subinvolution (blood deficiency, blood heat, and blood stasis), we did not class the formulae into those patterns for the incomplete information of most literature. Future research is needed to investigate the different medication rules based on dialectics.

## 5. Conclusions

This study explored the prescription laws of Chinese herbal medicinal formulae in the treatment of postpartum uterine subinvolution using integrated methods. A total of 803 formulae involving 249 herbs were obtained. The top 6 most frequently used herbs were *Angelicae Sinensis Radix* (Danggui), *Chuanxiong Rhizoma* (Chuanxiong), *Leonuri Herba* (Yimucao), *Persicae Semen* (Taoren), *Zingiberis Rhizoma Preparatum* (Paojiang), and *Radix Glycyrrhizae Preparata* (Zhigancao). Most of the 249 herbs were being warm in properties and sweet in tastes and were predominantly distributed to liver and spleen meridians. Among the 249 herbs, deficiency-tonifying herbs ranked the largest proportion and heat-clearing herbs ranked the second, followed by blood-activating and stasis-eliminating herbs. 5 clusters with clinical significance were obtained by hierarchical clustering, and 78 rules were obtained with support values over 0.25, confidence values over 0.8, and lift values greater than 1 by association rule learning.

The results of data mining revealed that the basic principles for uterine subinvolution treatment were deficiency-tonifying, heat-clearing, blood-activating, and stasis-eliminating. Herbs with warm properties, sweet tastes, and liver and spleen meridian tropisms are generally suitable for treatment. In addition, Sheng-Hua-Tang was the most frequently used formula for the treatment of uterine subinvolution, yet the dialectical prescriptions were diversified with different patterns/symptoms.

## Figures and Tables

**Figure 1:** Workflow of the literature search process for data mining.

**Figure 2:** Frequency chart of Chinese herbs treating uterine subinvolution. The top 30 most frequently used herbs were used for analysis.

**Figure 3:** Radar chart of properties, tastes, and meridian tropisms of the 249 herbs involved in all prescriptions. (a) Chart of properties. The warm, mild, cold, hot, and cool properties are represented by red, orange, green, light blue, and yellow dots, respectively. (b) Chart of tastes. The tastes of sweet, bitter, pungent, sour, salty, astringent, and weak are represented by red, orange, green, light blue, yellow, light gray, and blue, respectively. (c) Chart of meridian tropisms. The values of liver, spleen, heart, kidney, lung, stomach, large intestine, pericardium, gall bladder, bladder, tri-jiao, and small intestine are marked by red, orange, green, light green, light blue, purple, gray, dark golden, dark blue, dark orange, blue, and light orange dots, respectively.

**Figure 4:** Percentages of the number of herbs in different categories to the total number of herbs (249) treating uterine subinvolution.

**Figure 5:** Dendrogram of cluster analysis. The diagram was generated by IBM SPSS 26.0 software, and the top 40 most frequently used herbs were analyzed. C1∼C6 represent the 6 different clusters formed at the distance of 23, and the corresponding herbs were marked by different colors.

**Figure 6:** Chart of the 78 rules. (a) Item frequency chart. The top 10 frequent item sets. (b) Scatter plot. The *X*-axis represents the support level, and *Y*-axis represents the confidence level. The color of the dot represents the lift value, and the darker the color, the higher the lift value. (c) The network graph of 78 association rules. The size of circles indicates the confidence (0.802–1) level, and the color of circles indicates the lift (1.045–1.517) level.

**Figure 7:** The summary of prescription rules treating uterine subinvolution. The circles represent herbs involved. Herbs from different clusters were marked by different colored circles.

**Table 1:** Core herbs appeared over 48 times in prescriptions.

No.	Herb name	Frequency	Rate (%)
1	*Angelicae Sinensis Radix* (Danggui)	679	8.71
2	*Chuanxiong Rhizoma* (Chuanxiong)	586	7.51
3	*Leonuri Herba* (Yimucao)	554	7.10
4	*Persicae Semen* (Taoren)	509	6.53
5	*Zingiberis Rhizoma Preparatum* (Paojiang)	318	4.08
6	*Radix Glycyrrhizae Preparata* (Zhigancao)	310	3.97
7	*Astragali Radix* (Huangqi)	294	3.77
8	*Pollen Typhae* (Puhuang)	269	3.45
9	*Codonopsis Radix* (Dangshen)	245	3.14
10	*Glycyrrhizae Radix Et Rhizoma* (Gancao)	213	2.73
11	*Faeces Trogopteri* (Wulingzhi)	138	1.77
12	*Paeoniae Radix Alba* (Baishao)	136	1.74
13	*Atractylodes Macrocephala Rhizoma* (Baizhu)	134	1.72
14	*Paeoniae Radix Rubra* (Chishao)	133	1.71
15	*Rehmanniae Radix Praeparata* (Shudihuang)	129	1.65
16	*Aisni Corii Colla* (Ejiao)	124	1.59
17	*Flos Carthami* (Honghua)	106	1.36
18	*Crataegi Fructus* (Shanzha)	90	1.15
19	*Folium Artemisiae Argyi* (Aiye)	87	1.12
20	*Aurantii Fructus* (Zhike)	87	1.12
21	*Rehmanniae Radix* (Dihuang)	85	1.09
22	*Achyranthis Bidentatae Radix* (Niuxi)	84	1.08
23	*Dipsaci Radix* (Xuduan)	84	1.08
24	*Moutan Cortex* (Mudanpi)	76	0.97
25	*Cyperi Rhizoma* (Xiangfu)	69	0.88
26	*Poria Cocos (Schw*.*) Wolf*. (Fuling)	67	0.86
27	*Herba Taraxaci* (Pugongying)	65	0.83
28	*Bupleuri Radix* (Chaihu)	59	0.76
29	*Herba Patriniae* (Baijiangcao)	57	0.73
30	*Cyathulae Radix* (Chuanniuxi)	56	0.72
31	*Eucommiae Cortex* (Duzhong)	55	0.71
32	*Radix Sanguisorbae* (Diyu)	54	0.69
33	*Cinnamomi Cortex* (Rougui)	53	0.68
34	*Notoginseng Radix Et Rhizoma* (Sanqi)	53	0.68
35	*Rubia Cordifolia* (Qiancao)	52	0.67
36	*Rhizoma Dioscoreae* (Shanyao)	51	0.65
37	*Corydalis Rhizoma* (Yanhusuo)	49	0.63
38	*Zingiberis Rhizoma* (Ganjiang)	48	0.62
39	*Spatholobus Suberectus Dunn* (Jixueteng)	48	0.62
40	*Portulacae Herba* (Machixian)	48	0.62

**Table 2:** Action categories of herbs treating subinvolution of uterus.

Herb category	Frequency	Rate (%)
Deficiency-tonifying herbs	2685	34.43
Blood-activating and stasis-eliminating herbs	2338	29.98
Hemostatic herbs	1002	12.85
Heat-clearing herbs	722	9.26
Qi-regulating herbs	247	3.17
Superficies-relieving herbs	180	2.31
Interior-warming herbs	151	1.94
Dampness-draining diuretic herbs	102	1.31
Astringent herbs	88	1.13
Digestant herbs	97	1.24
Wind-damp dispelling herbs	57	0.73
Liver-wind calming herbs	26	0.33
Tranquilizing herbs	25	0.32
Purging herbs	23	0.29
Phlegm-dissolving and cough-asthma-relieving herbs	22	0.28
Dampness-resolving herbs	20	0.26
Antihelmintic herbs	7	0.09
Resuscitation-inducing herbs	4	0.05
Antitoxin, insecticide, and antipruritic herbs	3	0.04

**Table 3:** Association rules.

No.	Rules (antecedent⇒consequent)	Support	Confidence	Lift
1	{*Codonopsis Radix* (Dangshen)}⇒{*Angelicae Sinensis Radix* (Danggui)}	0.29	0.96	1.14
2	{*Pollen Typhae* (Puhuang)}⇒{*Leonuri Herba* (Yimucao)}	0.30	0.90	1.31
3	{*Pollen Typhae* (Puhuang)}⇒{*Chuanxiong Rhizoma* (Chuanxiong)}	0.27	0.81	1.11
4	{*Pollen Typhae* (Puhuang)}⇒{*Angelicae Sinensis Radix* (Danggui)}	0.30	0.90	1.07
5	{*Radix Glycyrrhizae Preparata* (Zhigancao)}⇒{*Persicae Semen* (Taoren)}	0.32	0.83	1.31
6	{*Radix Glycyrrhizae Preparata* (Zhigancao)}⇒{*Chuanxiong Rhizoma* (Chuanxiong)}	0.34	0.89	1.22
7	{*Radix Glycyrrhizae Preparata* (Zhigancao)}⇒{*Angelicae Sinensis Radix* (Danggui)}	0.37	0.96	1.14
8	{*Zingiberis Rhizoma Preparatum* (Paojiang)}⇒{*Persicae Semen* (Taoren)}	0.37	0.94	1.48
9	{*Zingiberis Rhizoma Preparatum* (Paojiang)}⇒{*Chuanxiong Rhizoma* (Chuanxiong)}	0.37	0.94	1.28
10	{*Zingiberis Rhizoma Preparatum* (Paojiang)}⇒{*Angelicae Sinensis Radix* (Danggui)}	0.39	0.98	1.16
11	{*Astragali Radix* (Huangqi)}⇒{*Angelicae Sinensis Radix* (Danggui)}	0.34	0.93	1.10
12	{*Persicae Semen* (Taoren)}⇒{*Chuanxiong Rhizoma* (Chuanxiong)}	0.58	0.91	1.25
13	{*Persicae Semen* (Taoren)}⇒{*Angelicae Sinensis Radix* (Danggui)}	0.62	0.98	1.16
14	{*Leonuri Herba* (Yimucao)}⇒{*Chuanxiong Rhizoma* (Chuanxiong)}	0.55	0.80	1.10
15	{*Leonuri Herba* (Yimucao)}⇒{*Angelicae Sinensis Radix* (Danggui)}	0.61	0.88	1.05
16	{*Chuanxiong Rhizoma* (Chuanxiong)}⇒{*Angelicae Sinensis Radix* (Danggui)}	0.72	0.99	1.17
17	{*Angelicae Sinensis Radix* (Danggui)}⇒{*Chuanxiong Rhizoma* (Chuanxiong)}	0.72	0.85	1.17
18	{*Leonuri Herba* (Yimucao), *Pollen Typhae* (Puhuang)}⇒{*Chuanxiong Rhizoma* (Chuanxiong)}	0.25	0.84	1.16
19	{*Chuanxiong Rhizoma* (Chuanxiong), *Pollen Typhae* (Puhuang)}⇒{*Leonuri Herba* (Yimucao)}	0.25	0.94	1.37
20	{*Leonuri Herba* (Yimucao), *Pollen Typhae* (Puhuang)}⇒{*Angelicae Sinensis Radix* (Danggui)}	0.28	0.92	1.09
21	{*Angelicae Sinensis Radix* (Danggui), *Pollen Typhae* (Puhuang)}⇒{*Leonuri Herba* (Yimucao)}	0.28	0.92	1.33
22	{*Chuanxiong Rhizoma* (Chuanxiong), *Pollen Typhae* (Puhuang)}⇒{*Angelicae Sinensis Radix* (Danggui)}	0.26	0.98	1.16
23	{*Angelicae Sinensis Radix* (Danggui), *Pollen Typhae* (Puhuang)}⇒{*Chuanxiong Rhizoma* (Chuanxiong)}	0.26	0.87	1.20
24	{*Leonuri Herba* (Yimucao), *Radix Glycyrrhizae Preparata* (Zhigancao)}⇒{*Persicae Semen* (Taoren)}	0.25	0.88	1.38
25	{*Persicae Semen* (Taoren), *Radix Glycyrrhizae Preparata* (Zhigancao)}⇒{*Chuanxiong Rhizoma* (Chuanxiong)}	0.30	0.95	1.30
26	{*Chuanxiong Rhizoma* (Chuanxiong), *Radix Glycyrrhizae Preparata* (Zhigancao)}⇒{*Persicae Semen* (Taoren)}	0.30	0.88	1.39
27	{*Persicae Semen* (Taoren), *Radix Glycyrrhizae Preparata* (Zhigancao)}⇒{*Angelicae Sinensis Radix* (Danggui)}	0.32	1.00	1.18
28	{*Angelicae Sinensis Radix* (Danggui), *Radix Glycyrrhizae Preparata* (Zhigancao)}⇒{*Persicae Semen* (Taoren)}	0.32	0.86	1.35
29	{*Leonuri Herba* (Yimucao), *Radix Glycyrrhizae Preparata* (Zhigancao)}⇒{*Chuanxiong Rhizoma* (Chuanxiong)}	0.27	0.94	1.29
30	{*Leonuri Herba* (Yimucao), *Radix Glycyrrhizae Preparata* (Zhigancao)}⇒{*Angelicae Sinensis Radix* (Danggui)}	0.28	0.97	1.15
31	{*Chuanxiong Rhizoma* (Chuanxiong), *Radix Glycyrrhizae Preparata* (Zhigancao)}⇒{*Angelicae Sinensis Radix* (Danggui)}	0.34	0.99	1.17
32	{*Angelicae Sinensis Radix* (Danggui), *Radix Glycyrrhizae Preparata* (Zhigancao)}⇒{*Chuanxiong Rhizoma* (Chuanxiong)}	0.34	0.91	1.25
33	{*Persicae Semen* (Taoren), *Zingiberis Rhizoma Preparatum* (Paojiang)}⇒{*Leonuri Herba* (Yimucao)}	0.30	0.81	1.17
34	{*Leonuri Herba* (Yimucao), *Zingiberis Rhizoma Preparatum* (Paojiang)}⇒{*Persicae Semen* (Taoren)}	0.30	0.94	1.49
35	{*Persicae Semen* (Taoren), *Zingiberis Rhizoma Preparatum* (Paojiang)}⇒{*Chuanxiong Rhizoma* (Chuanxiong)}	0.35	0.95	1.30
36	{*Chuanxiong Rhizoma* (Chuanxiong), *Zingiberis Rhizoma Preparatum* (Paojiang)}⇒{*Persicae Semen* (Taoren)}	0.35	0.95	1.49
37	{*Persicae Semen* (Taoren), *Zingiberis Rhizoma Preparatum* (Paojiang)}⇒{*Angelicae Sinensis Radix* (Danggui)}	0.37	0.99	1.18
38	{*Angelicae Sinensis Radix* (Danggui), *Zingiberis Rhizoma Preparatum* (Paojiang)}⇒{*Persicae Semen* (Taoren)}	0.37	0.95	1.50
39	{*Leonuri Herba* (Yimucao), *Zingiberis Rhizoma Preparatum* (Paojiang)}⇒{*Chuanxiong Rhizoma* (Chuanxiong)}	0.30	0.94	1.29
40	{*Chuanxiong Rhizoma* (Chuanxiong), *Zingiberis Rhizoma Preparatum* (Paojiang)}⇒{*Leonuri Herba* (Yimucao)}	0.30	0.81	1.17
41	{*Leonuri Herba* (Yimucao), *Zingiberis Rhizoma Preparatum* (Paojiang)}⇒{*Angelicae Sinensis Radix* (Danggui)}	0.31	0.98	1.16
42	{*Chuanxiong Rhizoma* (Chuanxiong), *Zingiberis Rhizoma Preparatum* (Paojiang)}⇒{*Angelicae Sinensis Radix* (Danggui)}	0.36	0.98	1.16
43	{*Angelicae Sinensis Radix* (Danggui), *Zingiberis Rhizoma Preparatum* (Paojiang)}⇒{*Chuanxiong Rhizoma* (Chuanxiong)}	0.36	0.94	1.29
44	{*Astragali Radix* (Huangqi), *Leonuri Herba* (Yimucao)}⇒{*Angelicae Sinensis Radix* (Danggui)}	0.28	0.95	1.13
45	{*Angelicae Sinensis Radix* (Danggui), *Astragali Radix* (Huangqi)}⇒{*Leonuri Herba* (Yimucao)}	0.28	0.81	1.18
46	{*Astragali Radix* (Huangqi), *Chuanxiong Rhizoma* (Chuanxiong)}⇒{*Angelicae Sinensis Radix* (Danggui)}	0.28	1.00	1.18
47	{*Angelicae Sinensis Radix* (Danggui), *Astragali Radix* (Huangqi)}⇒{*Chuanxiong Rhizoma* (Chuanxiong)}	0.28	0.83	1.14
48	{*Leonuri Herba* (Yimucao), *Persicae Semen* (Taoren)}⇒{*Chuanxiong Rhizoma* (Chuanxiong)}	0.45	0.94	1.29
49	{*Chuanxiong Rhizoma* (Chuanxiong), *Leonuri Herba* (Yimucao)}⇒{*Persicae Semen* (Taoren)}	0.45	0.80	1.27
50	{*Leonuri Herba* (Yimucao), *Persicae Semen* (Taoren)}⇒{*Angelicae Sinensis Radix* (Danggui)}	0.47	0.99	1.18
51	{*Chuanxiong Rhizoma* (Chuanxiong), *Persicae Semen* (Taoren)}⇒{*Angelicae Sinensis Radix* (Danggui)}	0.57	1.00	1.18
52	{*Angelicae Sinensis Radix* (Danggui), (Taoren)}⇒{*Chuanxiong Rhizoma* (Chuanxiong)}	0.57	0.93	1.27
53	{*Chuanxiong Rhizoma* (Chuanxiong), *Leonuri Herba* (Yimucao)}⇒{*Angelicae Sinensis Radix* (Danggui)}	0.55	0.99	1.17
54	{*Angelicae Sinensis Radix* (Danggui), *Leonuri Herba* (Yimucao)}⇒{*Chuanxiong Rhizoma* (Chuanxiong)}	0.55	0.90	1.24
55	{*Chuanxiong Rhizoma* (Chuanxiong), *Persicae Semen* (Taoren), *Radix Glycyrrhizae Preparata* (Zhigancao)}⇒{*Angelicae Sinensis Radix* (Danggui)}	0.30	1.00	1.18
56	{*Angelicae Sinensis Radix* (Danggui), *Persicae Semen* (Taoren), *Radix Glycyrrhizae Preparata* (Zhigancao)}⇒{*Chuanxiong Rhizoma* (Chuanxiong)}	0.30	0.95	1.31
57	{*Angelicae Sinensis Radix* (Danggui), *Chuanxiong Rhizoma* (Chuanxiong), *Radix Glycyrrhizae Preparata* (Zhigancao)}⇒{*Persicae Semen* (Taoren)}	0.30	0.89	1.41
58	{*Chuanxiong Rhizoma* (Chuanxiong), *Leonuri Herba* (Yimucao), *Radix Glycyrrhizae Preparata* (Zhigancao)}⇒{*Angelicae Sinensis Radix* (Danggui)}	0.26	0.98	1.16
59	{*Angelicae Sinensis Radix* (Danggui), *Leonuri Herba* (Yimucao), *Radix Glycyrrhizae Preparata* (Zhigancao)}⇒{*Chuanxiong Rhizoma* (Chuanxiong)}	0.26	0.95	1.30
60	{*Leonuri Herba* (Yimucao), *Persicae Semen* (Taoren), *Zingiberis Rhizoma Preparatum* (Paojiang)}⇒{*Chuanxiong Rhizoma* (Chuanxiong)}	0.28	0.95	1.30
61	{*Chuanxiong Rhizoma* (Chuanxiong), *Persicae Semen* (Taoren), *Zingiberis Rhizoma Preparatum* (Paojiang)}⇒{*Leonuri Herba* (Yimucao)}	0.28	0.80	1.17
62	{*Chuanxiong Rhizoma* (Chuanxiong), *Leonuri Herba* (Yimucao), *Zingiberis Rhizoma Preparatum* (Paojiang)}⇒{*Persicae Semen* (Taoren)}	0.28	0.95	1.49
63	{*Leonuri Herba* (Yimucao), *Persicae Semen* (Taoren), *Zingiberis Rhizoma Preparatum* (Paojiang)}⇒{*Angelicae Sinensis Radix* (Danggui)}	0.30	1.00	1.18
64	{*Angelicae Sinensis Radix* (Danggui), *Persicae Semen* (Taoren), *Zingiberis Rhizoma Preparatum* (Paojiang)}⇒{*Leonuri Herba* (Yimucao)}	0.30	0.81	1.17
65	{*Angelicae Sinensis Radix* (Danggui), *Leonuri Herba* (Yimucao), *Zingiberis Rhizoma Preparatum* (Paojiang)}⇒{*Persicae Semen* (Taoren)}	0.30	0.96	1.51
66	{*Chuanxiong Rhizoma* (Chuanxiong), *Persicae Semen* (Taoren), *Zingiberis Rhizoma Preparatum* (Paojiang)}⇒{*Angelicae Sinensis Radix* (Danggui)}	0.35	1.00	1.18
67	{*Angelicae Sinensis Radix* (Danggui), *Persicae Semen* (Taoren), *Zingiberis Rhizoma Preparatum* (Paojiang)}⇒{*Chuanxiong Rhizoma* (Chuanxiong)}	0.35	0.95	1.30
68	{*Angelicae Sinensis Radix* (Danggui), *Chuanxiong Rhizoma* (Chuanxiong), *Zingiberis Rhizoma Preparatum* (Paojiang)}⇒{*Persicae Semen* (Taoren)}	0.35	0.96	1.51
69	{*Chuanxiong Rhizoma* (Chuanxiong), *Leonuri Herba* (Yimucao), *Zingiberis Rhizoma Preparatum* (Paojiang)}⇒{*Angelicae Sinensis Radix* (Danggui)}	0.29	0.98	1.16
70	{*Angelicae Sinensis Radix* (Danggui), *Leonuri Herba* (Yimucao), *Zingiberis Rhizoma Preparatum* (Paojiang)}⇒{*Chuanxiong Rhizoma* (Chuanxiong)}	0.29	0.94	1.29
71	{*Angelicae Sinensis Radix* (Danggui), *Chuanxiong Rhizoma* (Chuanxiong), *Zingiberis Rhizoma Preparatum* (Paojiang)}⇒{*Leonuri Herba* (Yimucao)}	0.29	0.80	1.16
72	{*Chuanxiong Rhizoma* (Chuanxiong), *Leonuri Herba* (Yimucao), *Persicae Semen* (Taoren)}⇒{*Angelicae Sinensis Radix* (Danggui)}	0.44	1.00	1.18
73	{*Angelicae Sinensis Radix* (Danggui), *Leonuri Herba* (Yimucao), *Persicae Semen* (Taoren)}⇒{*Chuanxiong Rhizoma* (Chuanxiong)}	0.44	0.94	1.29
74	{*Angelicae Sinensis Radix* (Danggui), *Chuanxiong Rhizoma* (Chuanxiong), *Leonuri Herba* (Yimucao)}⇒{*Persicae Semen* (Taoren)}	0.44	0.81	1.28
75	{*Chuanxiong Rhizoma* (Chuanxiong), *Leonuri Herba* (Yimucao), *Persicae Semen* (Taoren), *Zingiberis Rhizoma Preparatum* (Paojiang)}⇒{*Angelicae Sinensis Radix* (Danggui)}	0.28	1.00	1.18
76	{*Angelicae Sinensis Radix* (Danggui), *Leonuri Herba* (Yimucao), *Persicae Semen* (Taoren), *Zingiberis Rhizoma Preparatum* (Paojiang)}⇒{*Chuanxiong Rhizoma* (Chuanxiong)}	0.28	0.95	1.30
77	{*Angelicae Sinensis Radix* (Danggui), *Chuanxiong Rhizoma* (Chuanxiong), *Persicae Semen* (Taoren), *Zingiberis Rhizoma Preparatum* (Paojiang)}⇒{*Leonuri Herba* (Yimucao)}	0.28	0.80	1.17
78	{*Angelicae Sinensis Radix* (Danggui), *Chuanxiong Rhizoma* (Chuanxiong), *Leonuri Herba* (Yimucao), *Zingiberis Rhizoma Preparatum* (Paojiang)}⇒{*Persicae Semen* (Taoren)}	0.28	0.96	1.52

**Table 4:** Characteristics of the top 40 herbs.

Categories		Herbs
Deficiency-tonifying herbs	Qi tonic	*Radix Glycyrrhizae Preparata* (Zhigancao), *Astragali Radix* (Huangqi), *Codonopsis Radix* (Dangshen), *Glycyrrhizae Radix Et Rhizoma* (Gancao), *Rhizoma Dioscoreae* (Shanyao), *Atractylodes Macrocephala Rhizoma* (Baizhu)
	Blood tonic	*Rehmanniae Radix Praeparata* (Shudihuang), *Aisni Corii Colla* (Ejiao), *Angelicae Sinensis Radix* (Danggui), *Paeoniae Radix Alba* (Baishao)
	Yang tonic	*Eucommiae Cortex* (Duzhong)
Blood-activating and stasis-eliminating herbs		*Chuanxiong Rhizoma* (Chuanxiong), *Achyranthis Bidentatae Radix* (Niuxi), *Leonuri Herba* (Yimucao), *Persicae Semen* (Taoren), *Faeces Trogopteri* (Wulingzhi), *Flos Carthami* (Honghua), *Dipsaci Radix* (Xuduan), *Cyathulae Radix* (Chuanniuxi), *Corydalis Rhizoma* (Yanhusuo), *Spatholobus Suberectus Dunn* (Jixueteng)
Hemostatic herbs		*Zingiberis Rhizoma Preparatum* (Paojiang), *Pollen Typhae* (Puhuang), *Aurantii Fructus* (Zhike), *Radix Sanguisorbae* (Diyu), *Notoginseng Radix Et Rhizoma* (Sanqi), *Rubia Cordifolia* (Qiancao)
Heat-clearing herbs		*Paeoniae Radix Rubra* (Chishao), *Rehmanniae Radix* (Dihuang), *Moutan Cortex* (Mudanpi), *Herba Taraxaci* (Pugongying), *Herba Patriniae* (Baijiangcao), *Portulacae Herba* (Machixian)
Qi-regulating herbs		*Folium Artemisiae Argyi* (Aiye), *Cyperi Rhizoma* (Xiangfu)
Superficies-relieving herbs		*Bupleuri Radix* (Chaihu)
Interior-warming herbs		*Cinnamomi Cortex* (Rougui), *Zingiberis Rhizoma* (Ganjiang)
Dampness-draining diuretic herbs		*Poria Cocos (Schw*.*) Wolf*. (Fuling)
Digestant herbs		*Crataegi Fructus* (Shanzha)

## Data Availability

All data used to support the findings of this study are included within the article.

## Abbreviations

PPH: Secondary postpartum hemorrhage
CNKI: China National Knowledge Infrastructure Database
CBM: Chinese Biomedical Literature Database
VIP: Database of Chinese Technical Periodicals
WanFang: WanFang data
TCM: Traditional Chinese medicine.
